RETRACTED

# Response to: “Questioning the evidence for BCI-based communication in the complete locked-in state”

**DOI:** 10.1371/journal.pbio.3000063

**Published:** 2019-04-08

**Authors:** Ujwal Chaudhary, Sudhir Pathak, Niels Birbaumer

**Affiliations:** 1 Institute of Medical Psychology and Behavioral Neurobiology, Eberhrd-Karls University of Tuebingen, Tuebingen, Germany; 2 Wyss Center for Bio and Neuroengineering, Geneva, Switzerland; 3 Learning Research and Development Center (LRDC), University of Pittsburgh, Pittsburgh, United States of America; Charite Universitatsmedizin Berlin, GERMANY

Patients in completely locked-in state (CLIS) have no means of communication and present a highly challenging and daunting problem for the neuroscientist [1–3]. Until today, few groups have attempted to solve this problem, and only some have reported success in advancing the goal of providing a means of communication to patients in CLIS [4–7]. In his commentary, Dr. Spüler raises doubts about all the research efforts towards this goal but primarily about the results published in 2017 by Chaudhary and colleagues. Dr. Spüler bases the commentary on 2 main calculations:

1. Absence of hemodynamic differences between “yes” and “no” thinking and
2. Chance-level classification across all the sessions in the 4 published cases with CLIS.

In this commentary, we address the issues raised by Dr. Spüler.

## 1. Absence of hemodynamic differences between “yes” and “no” thinking

In his commentary, Dr. Spüler claims that, in the paper by Chaudhary and colleagues [6], the change in the concentrations of oxy-hemoglobin (O_2_Hb) acquired from 20 different functional near-infrared spectroscopy (fNIRS) channels were averaged, and then further averaging was performed across trials and sessions. Chaudhary and colleagues [6] presented the averaged change in relative concentration of O_2_Hb separately for each of the 20 channels used during the study, as shown in their Fig 1 [6]. In none of the fNIRS literature published to date have fNIRS channels placed across such disparate regions been averaged [8–12]. The reason behind not averaging the channels is the fact that different channels represent metabolic information from the respective underlying brain region. In Chaudhary and colleagues’ paper [6], therefore, first signal acquired across different trials—i.e., “yes” and “no” thinking—were averaged separately for the different channels and were then averaged across sessions as shown in Fig 1 of Chaudhary and colleagues [6]. Fig 1 of Chaudhary and colleagues’ paper shows the averaged relative change in O_2_Hb from all the 20 channels; if all 20 channels were averaged, then we would have had just 1 time-series of relative change in O_2_Hb and not 20 different time-series of relative change in O_2_Hb, each corresponding to a channel, as depicted by Chaudhary and colleagues. To further elucidate the difference in hemodynamic response between “yes” and “no” thinking, general linear model (GLM) analysis was performed as shown in S1 Text. Dr. Spüler’s claim of a lack of difference between the 2 response categories “yes” and “no” thinking is thus unfounded and not comparable to that of Chaudhary and colleagues. As reported by Chaudhary and colleagues, channels were treated separately for classification and model building for online feedback session as written on page 18 and 19 of Chaudhary and colleagues’ paper. According to Chaudhary and colleagues (page 18), “The mean of relative change in O_2_Hb across each channel was used as a feature to train the SVM model through a 5-fold cross-validation procedure.” On page 19, Chaudhary and colleagues further state that, “During an online feedback session, fNIRS data acquired online corresponding to each ISI was processed to obtain the relative change in O_2_Hb, as described above, across all the channels. The mean of the relative change in O_2_Hb across all the channels was used as test feature to map onto model space.”

RETRACTED

**Fig 1:** Bar graph of offline classification accuracy results obtained from the sessions performed by the patient B and published by Chaudhary and colleagues [6]. (A) The offline classification accuracy of sessions performed by patient B using the method reported by Chaudhary and colleagues, i.e., the mean O_2_Hb response was used as input feature for the linear support vector machine classifier. (B) The offline classification accuracy of sessions performed by patient B using the method suggested by Martin Spüler. (C) The offline classification accuracy of sessions performed by patient B using the CSP for feature extraction and using linear SVM classifier. CSP, common spatial pattern; O_2_Hb, oxy-hemoglobin; SVM, support vector machine.

## 2. Chance-level classification across all the sessions

Spüler raises doubts about the classification results based on the method he employed to calculate the offline classification accuracy of each session. It is well known in the machine learning literature that application of different machine learning algorithms and features results in different outcomes, as is obvious from the result presented by Dr. Spüler. We can argue on the method that can and should be used for classification, but that does not invalidate the results presented by Chaudhary and colleagues [6]. It has also been argued that the sessions should be combined randomly to build a model; we argue that such a method might be valid for stable and invariant data but might be completely misleading for patients in CLIS. As reported by Chaudhary and colleagues, physiological and psychological states (arousal and attention) of the patients should be considered when performing the analysis because these patients spend long periods of the waking day sleeping and dozing, hence only sessions during which patients were vigilant should be used to build classification models to provide feedback to the patients. Therefore, combining sessions randomly to build the classification model would include time periods of an unresponsive state of the particular patient. The correlations of electroencephalogram (EEG) slow activity with performance, we reported in the original paper, underscore this point and demonstrate that such a relationship with lack of arousal and poor performance exists. These issues were thoroughly discussed in the section entitled “Slow EEG rhythms’ relationship with fNIRS classification accuracy” on page 8 as well as the discussion section on page 12 titled “BCI performance and attention-vigilance” of Chaudhary and colleagues’ paper. Thus, Dr. Spüler’s failure to replicate our results may originate from such a random treatment and random selection of sessions to calculate the classification precisions of patients’ mental answers. Assuming that we continue a session on a day when the patient is unresponsive, the EEG shows dominant slow-wave activity of 1 to 2 Hz, and we build the model to perform online feedback session—in such a case, the patient will receive wrong feedback over an extended time period not determined by his or her actual performance but by an episode of deep sleep and unresponsiveness.

RETRACTED

Here, we present the classification result using the data from patient B from 3 different analysis methods, as follows: (a) the method described by Chaudhary and colleagues (shown in Fig 1A), (b) the method proposed by Martin Spüler (shown in Fig 1B), and (c) using common spatial pattern (CSP) [13] (details shown in S1 Text) to extract the feature and then performing classification (shown in Fig 1C).

Thus, based on the result presented in this section, it can be seen that we can implement different methods, which can have both negative and positive effect on classification result. The goal of our ongoing research is to find and apply the best strategy to improve the classification accuracy to increase the overall communication rate with patients [14], which we have stated clearly in the discussion section of Chaudhary and colleagues’ paper.

## Slowing of EEG and consciousness

Slowing of EEG frequencies as found in many CLIS patients with amyotrophic lateral sclerosis (ALS) and other neurological conditions can have many reasons, such as the simple fact that these patients have to use artificial ventilation, which bypasses breathing through the nose. The neuronal epithelium involved in olfaction synchronizes high frequency (beta and gamma) in the entire brain of mammals [15]. Thus, slowing of frequencies may just indicate a side effect of bypassing airflow from nose to the trachestoma and not any “impaired cognitive abilities.” Martin Spüler continues, in his discussion, to question the cognitive intactness of CLIS patients, claiming that alpha wave indicates “consciousness” and suggesting implicitly that their absence points to a lack of conscious processing. Such a claim is not only wrong but also medically dangerous because of attribution of conscious experience to unconscious patients and frequent misdiagnoses. In addition, alpha waves are not a unitary concept but a general term for very heterogeneous physiological phenomena: alpha of the sensorimotor cortex, for example—also called somatosensory alpha or sensorimotor rhythm [16] or mu rhythm—indicates quiescence of the motor system, with no relationship to any form of consciousness. Auditory alpha exclusively originating from the central auditory cortex is interpreted as an inhibitory state of the central auditory analysis—again, no relationship with consciousness. An extensive literature [17] on visual, occipital alpha waves has shown that their presence depends heavily on coupling and uncoupling of the oculomotor system, which is a purely motor phenomenon independent of the conscious state of the organism. Comprehensive discussion and information of the physiological basis of alpha rhythm can be found in Andersen and Andersson [18] and Klimesch and colleagues [19]. Moreover, patients in Chaudhary and colleagues’ publication participated in some of these testing procedures [20], and all showed an electrophysiological correlate of cognitive processing (not presented in Chaudhary and colleagues’ 2017 paper, as that was not the goal of the paper).

RETRACTED

## Missing data link

https://doi.org/10.5281/zenodo.1419151

We committed an error in uploading the data of patient F: we uploaded the data of 28 sessions, although Chaudhary and colleagues contain the results of 58 sessions from patient F. Herein, we are uploading the remaining data from this patient, whose results are already included in the Chaudhary and colleagues’ paper.

## Supporting information

S1 Text “Yes” and “no” thinking, GLM analysis, and classification using CSP. (DOCX)

S1 Fig Difference in hemodynamic response between “yes” and “no” thinking using general linear model. (TIFF)

S2 Fig Binary map of the *t* test between “yes” and “no” thinking. (TIFF)

## Abbreviations

ALS: amyotrophic lateral sclerosis
CLIS: completely locked-in state
CSP: common spatial pattern
EEG: electroencephalogram
fNIRS: functional near-infrared spectroscopy
GLM: general linear model
O_2_Hb: oxy-hemoglobin
